The article "The Value of High-Resolution Ultrasound Combined with Shear-Wave Elastography under Artificial Intelligence Algorithm in Quantitative Evaluation of Skin Thickness in Localized Scleroderma" was published in 2022. Journal: Comput Intell Neurosci.

# The Value of High-Resolution Ultrasound Combined with Shear-Wave Elastography under Artificial Intelligence Algorithm in Quantitative Evaluation of Skin Thickness in Localized Scleroderma

**DOI:** 10.1155/2022/1613783

**Published:** 2022-03-04

**Authors:** Kun Jia, Huiying Li, Xiaojing Wu, Caina Xu, Hongyuan Xue

**Affiliations:** Department of Ultrasound, Hebei General Hospital, Shijiazhuang, Hebei 050000, China

## Abstract

The aim of this study was to explore the value of high-resolution ultrasound combined with shear-wave elastography (SWE) in measuring skin thickness in patients with localized scleroderma (LS). Fifty patients with LS diagnosed by pathology in the hospital were selected as the research object, with a total of 96 lesions. Healthy people (50 cases) in the same period were selected as the control group. The skin thickness of the abdomen, chest, and left finger of the two groups was compared. The traditional nonlocal means (NLM) algorithm was improved by changing the Euclidean distance and introducing a cosine function, which was applied to the ultrasonic imaging intelligent diagnosis of patients with localized scleroderma. SWE imaging was evaluated, and the results demonstrated that LS lesion edema stage accounted for 7.29%, hardening stage occupied 43.75%, and the proportion of atrophy stage reached 48.96%. When the size of shell was 1 mm, maximum elastic modulus (*E*_max_) was 0.984, mean of elastic modulus (Emean) was 0.926, and electro-static discharge (Esd) was 0.965. When the size of shell was 2 mm, the elastic moduli around lesions were as follows: Emax was 0.998, Emean was 0.968, and Esd was 0.997. By comparing the skin thickness of the abdomen, chest, and left finger, it was found that there was a significant difference between the LS group and the control group (*P* < 0.05). When the shell was 2 mm, the effect of sensitivity specificity on SWE imaging was better than that when the shell was 1 mm. In summary, the improved NLM algorithm showed excellent denoising effects on the ultrasonic images of LS patients. Besides, it could assist clinicians in ultrasonic imaging diagnosis for LS patients and effectively improve the diagnostic accuracy of diseases.

## 1. Introduction

Scleroderma is a connective tissue disease characterized by skin inflammation, degeneration, thickening, fibrosis, and then, hardening and atrophy [1]. Localized scleroderma (LS) is characterized by primary skin and subcutaneous fibrosis. The pathogenesis of LS is related to many reasons, including activation and imbalance of the immune system, changes of small blood vessels in the dermis, and fibroblast activation and fibrosis [2–4]. The treatment principle of scleroderma skin hardening and thickening is early diagnosis and early treatment, which can help to prevent disease progression [5, 6]. The degree of skin fibrosis in patients with LS is closely related to the clinical stage of the disease and visceral involvement. Ultrasound can accurately detect nerve continuity, echo, and mobility. However, the quantitative indexes measured by ultrasound have a poor correlation with nerve repair status, and the clinical application is limited [7, 8]. In addition, there are also operator dependence, semiquantitative skin thickness evaluation, and insensitive to some small changes. High-frequency ultrasound is one of the high-resolution imaging tools. It is widely used in the clinical evaluation of skin thickness [9, 10]. It has been shown by some scholars that the quantification of skin thickness by high-frequency ultrasound has the characteristics of good repeatability, objectivity, and reliability [11].

The article "The Value of High-Resolution Ultrasound Combined with Shear-Wave Elastography under Artificial Intelligence Algorithm in Quantitative Evaluation of Skin Thickness in Localized Scleroderma" was published in 2022. Journal: Comput Intell Neurosci.

Shear-wave elastography (SWE) is a new technology and developed rapidly in recent years. It can quantitatively evaluate tissue hardness. The emergence of this technology breaks the limitations of conventional anatomical results imaging [12, 13]. SWE has the advantages of noninvasive and convenient quantification. The imaging system is mainly based on the trial excitation of the tissue by emitting acoustic radiation pulses. The counting core generates shear waves with sufficient strength in the tissue according to the principle of “Mach vertebra”. The ultrahigh-speed imaging technology is used to detect shear waves with an accuracy of more than 1nm/s [14, 15]. Nonlocal means (NLM) denoising algorithm mainly uses self-similar structural blocks as weighted average to estimate the center point of the reference block, so as to reduce noise (Gaussian white noise with zero mean). NLM has good denoising effect [16, 17]. At present, two-dimensional ultrasonography is the most widely used in the clinic, with clear boundary, strong operability, and good patient compliance. Semiannular or annular color blood flow signals can be observed under color Doppler ultrasound. At present, two-dimensional B-ultrasound is the main ultrasonic diagnosis technology in China. Ultrasound has various characteristics of sound waves. In the process of ultrasonic propagation, ultrasound passes through tissues and organs with different structures, resulting in different degrees of attenuation. The receiving end receives echoes of different degrees. After marking with light spots with different gray levels on the shadow screen, the sectional imaging of the tested organ or tissue is obtained [18, 19]. However, complex ultrasonic image features can be observed in the process of ultrasonic diagnosis and are affected by ultrasonic detection technology and its imaging mechanism. Noise will inevitably be produced because of the mutual interference of many ion beams and the scattering and superposition of echo signals. The emergence of noise affects clinicians' observation of medical images to a certain extent and even leads to the misdiagnosis of diseases. In the process of ultrasound imaging, the NLM algorithm is applied to intelligently remove the speckle noise in imaging, which is conducive to improving the clarity of ultrasound. Shear-wave ultrasound imaging has many clinical studies on the hardness of the breast, liver, thyroid, and other tissues. Compared with the weighted average in global search by bilateral-filtering NLM denoising algorithm, the replacement of the distance between pixels by weighted Euclidean distance between image blocks shows excellent denoising ability and can better retain the structural information of images, including points and lines. The combination of the NLM algorithm with ultrasonic SWE can offer images with a higher level of definition and enhance the diagnostic efficiency of skin diseases. Ultrasonic elastography refers to the production of corresponding strain, displacement, or velocity distribution in tissues under the physical laws of elasticity or biomechanics. The combination of ultrasonic imaging and digital algorithm technology can help estimate the strain and displacement parameters inside tissues and further directly or indirectly reflect the differences in elastic modulus and other mechanical properties. At present, there are few reports on the application of ultrasonic shear-wave elastography in the evaluation of skin thickness in localized scleroderma.

The article "The Value of High-Resolution Ultrasound Combined with Shear-Wave Elastography under Artificial Intelligence Algorithm in Quantitative Evaluation of Skin Thickness in Localized Scleroderma" was published in 2022. Journal: Comput Intell Neurosci.

In this study, the NLM algorithm is applied to the image analysis and diagnosis of patients with high-resolution ultrasound combined with shear-wave elastic imaging. SWE detection is applied in the diagnosis of skin hardness disease, which offers a new direction to the characterization study on elastic tissues. Besides, the clinical application of shear-wave quantitative elastography technology in scleroderma is discussed.

The misjudgment rate of diagnosis can be effectively reduced in this way. By discussing the application value of ultrasonic shear-wave elastic imaging technology in the skin thickness of localized scleroderma, it is expected to provide new ideas for the quantitative evaluation of scleroderma in the clinic. Moreover, it is expected to do a great contribution to the improvement of patients' quality of life.

## 2. Methods and Materials

### 2.1. Cases

Fifty patients with LS diagnosed by pathology in the hospital were selected as the research object, with a total of 96 lesions (LS group). This study was approved by the medical ethics committee of the hospital, and all the patients signed the informed consent.

The article "The Value of High-Resolution Ultrasound Combined with Shear-Wave Elastography under Artificial Intelligence Algorithm in Quantitative Evaluation of Skin Thickness in Localized Scleroderma" was published in 2022. Journal: Comput Intell Neurosci.

The pathological changes were discussed according to pathological stages (hardening stage, edema stage, and atrophy stage). High-frequency ultrasound combined with shear-wave elasticity was used to measure the skin hardness and thickness of LS lesions and unaffected parts around the contralateral side, which were selected as normal controls. The differences of lesion sites were compared according to normal skin thickness and elastic modulus (*E*). The relative difference of skin elastic modulus (M_RD_) between lesions and normal controls was analyzed, and then, the differences of relative values between different case stages were compared. There were no significant differences in age, gender, and other general data between research objects in two groups (*P* > 0.05) but comparability.

Inclusion criteria were as follows: all patients were clearly diagnosed by LS and had good compliance. The inclusion criteria of the control group were healthy persons (50 cases) in the same period. Exclusion criteria were as follows: other skin diseases, combined with rheumatic immune diseases, history of radiotherapy, and history of endocrine metabolic emergencies.

### 2.2. Ultrasonic Elastography

Elastic imaging was born 20 years ago. Tissue hardness was a powerful index related to the normality of tissue. Elastic imaging was of great significance for clinical tissue hardness evaluation. It was an important factor to improve the noninvasive, sensitivity, and reliability of clinical tissue hardness evaluation. The ultimate purpose of ultrasonic elastic imaging was to provide information about the mechanical properties of tissue, mainly Young's Modulus, that is, the hardness of tissue. The hardness of tissue was expressed by Young's Modulus, and the mechanical properties of tissue were evaluated quantitatively. The classification and induction of ultrasonic elastic imaging methods are illustrated in Figure 1.

### 2.3. NLM Algorithm Image Processing

The core of the image denoising algorithm was to use the algorithm to process the image to obtain a similar result to the image without noise interference. It was assumed that the image without noise was *O*_*i*_ and the noise was *N*_*i*_, and the mathematical model of the denoised image can be set as *O*_*i*_′=*O*_*i*_+*N*_*i*_. In the actual process, there are many algorithms used for image filterings, such as mean filtering, median filtering, Gaussian filtering, and bilateral filtering.

The article "The Value of High-Resolution Ultrasound Combined with Shear-Wave Elastography under Artificial Intelligence Algorithm in Quantitative Evaluation of Skin Thickness in Localized Scleroderma" was published in 2022. Journal: Comput Intell Neurosci.

The NLM algorithm is a kind of algorithm that uses the redundant information of the image in the pixel or spatial domain to remove image noise without destroying the edge features of the image. It was assumed in this work that the target image was y(x), and the uncorrelated additive white Gaussian noise was n(x), and then, the noise image was f(x) = *y*(x) + *n*(x). The NLM algorithm was used to search and compare the gray value of the pixels in the noise image f(x) and analyze the similarity of the pixels in the target area and the field, so as to obtain the weighted average to remove the noise in the image. The target pixel was set as the center, the search window was set, and the similarity of adjacent windows was compared by narrowing the search range to obtain the weight value. Therefore, the mathematical model of image filtering processing using the NLM algorithm can be defined as

(1) $$\begin{array}{c} NLM\left[a\right]\left(i\right)=\frac{1}{\sigma \left(i\right)}\cdot \sum_{j\in G}w\left(i,j\right)a\left(j\right). \end{array}$$

In (1), *NLM[a](i)* was the value of the target pixel after weighted average processing, *G* was the gray value, *i* was the target pixel, *j* referred to an arbitrary pixel, *σ(i)* represented the normalization constant, and *w(i, j)* was the similarity between the target pixel and the domain window of neighboring pixels.

(2) $$\begin{array}{c} w\left(i,j\right)=\frac{1}{\alpha \left(i\right)}\cdot \text{exp}\left[-d\frac{\left(i,j\right)}{\mu }\right]. \end{array}$$

In (2), *α(i)* was the normalization constant, *d(i, j)* represented the Euclidean distance weighted by Gaussian, and *μ* referred to the filtering parameter of the image smoothness.

The basic flow of ultrasonic image denoising processing using the NLM algorithm is shown in Figure 2.

In order to improve the performance of the NLM algorithm, the regularization model was adopted in this work to optimize the NLM algorithm. The output image was assumed as *u*, and the predicted image was assumed as *v*, so the Bayesian maximum posterior probability of the image can be set as follows:

(3) $$\begin{array}{c} u_{\text{map}}=\text{max}\frac{\left[P\left(v|u\right)P\left(u\right)\right]}{P\left(v\right)}. \end{array}$$

In (3), *P*(*v|u*) was the probability of occurrence of *v* under the condition of *u*.

ADMM was introduced to optimize the solution of the improved algorithm, so equation (2) can be rewritten as

(4) $$\begin{array}{c} u_{\text{map}}=\text{min}\left\{-\text{log}\left[P\left(v|u\right)\right]-\text{log}\left[P\left(u\right)\right]\right\}. \end{array}$$

Then, the image denoising was introduced, and the adaptive Laplacian operator was used to solve equation (3), so as to obtain the final optimized and improved NLM algorithm.

(5) $$\begin{array}{c} E\left(u\right)=\frac{1}{2\alpha^{2}}Hu-v_{2}^{2}+\frac{\beta }{2}u^{T}\left[u-NLM\left(u\right)\right],\\ \left\{u_{\text{map}},y^{\prime },x^{\prime }\right\}=\text{min}h\left(v,u\right)+\beta n\left(y\right)+\frac{\delta }{2}u-y+x_{2}^{2}. \end{array}$$

In the above equation, *δ* needed to be determined according to the noise level, *x* was the constraint of the Lagrange multiplier vector, and *β* = 0.02.

The article "The Value of High-Resolution Ultrasound Combined with Shear-Wave Elastography under Artificial Intelligence Algorithm in Quantitative Evaluation of Skin Thickness in Localized Scleroderma" was published in 2022. Journal: Comput Intell Neurosci.

### 2.4. Ultrasonic Measurement

A digital color Doppler ultrasound diagnostic instrument was used. The instrument possessed a real-time shear-wave elastic imaging function, and the probe frequency was 4–15MHz. SWE was measured by the ultrasonic detector, with linear array probe and frequency of 3–10MHz. The patient's skin was smeared with sufficient coupling agent and gently placed on the skin surface. The skin of the part to be tested shall be fully exposed. After routine disinfection, the thickness of the lesion and the skin of the normal part shall be measured by high-frequency ultrasound under the lowest pressure. The image shall be frozen after 3–5 seconds. The subject shall be instructed to hold his breath. The elastic diagram of each lesion shall be recorded, and the dynamic video frequency shall be stored in the ultrasonic instrument for analysis and interpretation by the doctor. The data and image were stored in the image, and the same part was measured for three consecutive times to take the average value. The operation process of shear-wave ultrasonic elastography was completed independently by two ultrasonic diagnostic physicians to ensure that the whole process was not interfered with each other.

Ultrasonic elastic images were acquired by real-time shear-wave elasticity direct quantization imaging technology, and the time-domain composite autocorrelation strain measurement method was selected and utilized. The shear wave was related to the elasticity of tissues. The hardness of tissues was expressed by elastic modulus *E*, which was the ratio of unconnected pressure (S) to tissues strain (e), and the calculation equation was *E* = *S*/*e*. Shear-wave elastic images were performed with color encoding and then superimposed on two-dimensional gray-scale diagrams. The harder images were shown in red, and the softer images were marked in blue.

Three elastic maps were selected from the scanned images to measure the elastic modulus of the region of interest, and the quantitative analysis was conducted on whether there was a “hard ring sign” in the lesion location. The edge of the lesion could be outlined. According to the interface displayed by the system, the “shell” function key was pressed to adjust the shell size, namely, to obtain the elastic modulus value of the 1 mm area outside the lesion boundary. The system automatically calculated the elastic modulus values, *E*_max_, Esd, *E*_min_, and Emean. The basic clinical data of the subject shall be informed to the physician before the evaluation.

The article "The Value of High-Resolution Ultrasound Combined with Shear-Wave Elastography under Artificial Intelligence Algorithm in Quantitative Evaluation of Skin Thickness in Localized Scleroderma" was published in 2022. Journal: Comput Intell Neurosci.

### 2.5. Diagnostic Evaluation

In this work, mean squared error (MSE), peak signal-to-noise ratio (PSNR), and structural similarity (SSIM) were used to evaluate the denoising effect of the NLM algorithm. The calculation equations of different evaluation indicators were as follows:

(6) $$\begin{array}{c} MSE=\frac{1}{\left(mn\right)}\cdot \overset{m-1}{\underset{i=0}{\sum }}\sum_{j=0}^{n-1}I\left(i,j\right)-K{\left(i,j\right)}^{2}. \end{array}$$

In the equation above, *m* and *n* represented the pixel position of the same size image, and *I* and *K* both represented the image whose mean square error needs to be calculated. When the MSE value is smaller, the denoised image is closer to the undisturbed image, and the filtering effect of the algorithm is better.

(7) $$\begin{array}{c} PSNR=10{\text{log}}_{10}\left(\frac{L^{2}}{MSE}\right). \end{array}$$

In equation (7) above, *L* represented the maximum pixel value in the search range. The larger the PSNR value, the less noise in the denoised image, and the better the filtering effect of the algorithm.

(8) $$\begin{array}{c} \text{SSIM}=\frac{\left(2\mu_{i}\mu_{j}+c_{1}\right)\left(\sigma_{ij+}c_{2}\right)}{\left(\mu_{i}^{2}+\mu_{j}^{2}+c_{1}\right)\left(\sigma_{i}^{2}+\sigma_{j}^{2}+c_{2}\right)}. \end{array}$$

In the above equation, *c* was a constant, *i* and *j* were the original image and the undisturbed image, *μ* represented the average of *i* and *j*, and *σ* referred to the covariance of *i* and *j*.

### 2.6. Statistical Processing Methods

The statistical software SPSS 20.0 was used for data analysis. It conformed to the normal distribution. The measurement data were expressed by mean ± standard deviation. The measurement data were normally distributed and had uniform variance. The sample mean comparison adopted an independent sample *t*-test. Nonparametric superposition test was used to compare the data groups with non-normal distribution and uneven variance. *P* < 0.05 was statistically significant.

## 3. Results

### 3.1. Comparison of Ultrasonic Images before and after Algorithm

NLM noise reduction algorithm had a certain inhibitory effect on the noise of patients' ultrasonic images. The improved NLM algorithm used in this study had a visual effect on the noise reduction of patients' ultrasonic images. The improved NLM algorithm had a certain effect on the noise reduction of patients' ultrasonic images, whether in terms of smoothness, detail retention, or accuracy of detail judgment.  Figure 3 reveals the ultrasonic diagram before the algorithm and the ultrasonic diagram for noise reduction of the NLM algorithm.

The article "The Value of High-Resolution Ultrasound Combined with Shear-Wave Elastography under Artificial Intelligence Algorithm in Quantitative Evaluation of Skin Thickness in Localized Scleroderma" was published in 2022. Journal: Comput Intell Neurosci.

Then, the indicators MSE, PSNR, and SSIM were used to objectively evaluate the effect of ultrasonic image denoising with the NLM algorithm before and after the improvement. The results are shown in Figure 4. With the increase of noise standard deviation, the MSE value of NLM and the improved NLM algorithm gradually increased, while the PSNR and SSIM values gradually decreased. Under different noise standard deviations, the MSE value of the improved NLM algorithm proposed was always smaller than the NLM algorithm, while the PSNR and SSIM values were larger than the NLM algorithm.

### 3.2. Ultrasonic Focus Map

Figure 5 indicates the outline of the edge of the lesion. Figure 5(a) shows the elastic modulus around the lesion when the shell was taken as 1 mm, as illustrated in Table 1, Emax is 0.984, Emean is 0.926, and Esd is 0.965. Figure 5(b) suggests the elastic modulus around the lesion when the shell was taken as 2 mm, Emax is 0.998, Emean is 0.968, and Esd is 0.997. AUC (area under curve) was the area surrounded by the coordinate axis under the ROC curve.

### 3.3. SWE Imaging Evaluation

The sensitivity specificity is illustrated in Figure 6 when the shell was 1 mm and 2 mm, and the diagnostic efficiency was better when the shell was 2 mm. The ROC curve of the shell with 1 mm elastic modulus is presented in Figure 7, Emax was greater than Emean, and the ROC curve of shell with 2 mm elastic modulus is presented in Figure 8. The effects of Emax were superior to those of Emean.

### 3.4. Statistical Results of LS Lesions

There were 96 lesions (as illustrated in Table 2), including 7 cases in the edema stage, 42 cases in the sclerosis stage, and 47 cases in the atrophy stage. The edema stage was not statistically analyzed. This study mainly focused on the hardening stage. Compared with normal skin, the elastic modulus of LS lesions in the sclerotic and atrophic stage was greater than that of normal control skin. The thickness in the atrophic stage was smaller. After correction of skin elastic modulus, the thickness in the sclerotic stage increased by 51.3% compared with that in the control stage.

### 3.5. Skin Thickness Comparison

The comparison of skin thickness in different parts is illustrated in Figure 9. The skin thickness of the abdomen, chest, and left finger of the two groups was compared. The results showed that there was a significant difference between the LS group and the control group (*P* < 0.05).

The article "The Value of High-Resolution Ultrasound Combined with Shear-Wave Elastography under Artificial Intelligence Algorithm in Quantitative Evaluation of Skin Thickness in Localized Scleroderma" was published in 2022. Journal: Comput Intell Neurosci.

## 4. Discussion

Scleroderma was a rare disease with two main forms: localized scleroderma (LS) and systemic sclerosis (SSc). Both were chronic diseases that could occur in different patterns (subtypes) and were related to the extracutaneous involvement of pediatric patients. The incidence rate and mortality rate of SSc patients with life-threatening lung, heart, and other internal organs fibrosis and vascular diseases were much lower. The mortality rate of LS was very low, but the incidence rate was high. Patients were at risk of severe disfigurement and dysfunction. The treatment of scleroderma was aimed at controlling inflammation and managing specific problems. Early diagnosis could greatly improve the results. Localized scleroderma was a disease characterized by localized skin fibrosis. At present, there was no unified evaluation standard. Many evaluation methods were applied in the treatment of this disease, such as computer scoring and semiquantitative scoring. Laser Doppler flowmetry, magnetic resonance, and ultrasound were applied in LS disease. The main treatment of localized scleroderma was still focused on antifibrosis and immune regulation. Zulian et al. (2007) [20] calculated the standard score of skin lesion area and overall surface area by using hard skin lesion edge tracing and transparent film. This was conducive to the development of patients' condition, but it was difficult to measure in uneven positions. Mamontov et al. (2020) [21] used the instrument identification of proximal scleroderma for the early diagnosis of systemic sclerosis. Imaging photoplethysmography (IPPG) had potential diagnostic value in evaluating systemic sclerosis.

Ultrasonic elastic imaging technology could individually quantify the elastic characteristics of a single skin layer. It was also a new technology used to study the elastic information of biological tissue in recent years. It could provide comprehensive skin information but could not provide skin thickness information. High-frequency ultrasound could measure the thickness of the skin. Many studies also confirmed its effectiveness and reliability [9]. NLM algorithm could make full use of redundant information in the image to reduce noise and fully retained the key information of the image. However, the NLM algorithm had high time complexity. There were still some artifacts in the denoised image, and there may be a risk of image information loss when the image filtering coefficient was large [22]. During the image processing of patients, the spatial position difference of lesion edge, vascular trunk, and other parts made it difficult for the similarity weight of the NLM algorithm to fully identify the similarity of pixel blocks. This led to insufficient image noise reduction. Thus, the algorithm was improved [23].

The article "The Value of High-Resolution Ultrasound Combined with Shear-Wave Elastography under Artificial Intelligence Algorithm in Quantitative Evaluation of Skin Thickness in Localized Scleroderma" was published in 2022. Journal: Comput Intell Neurosci.

According to the differences between image blocks rather than spatial distance, the NLM algorithm calculates the weight coefficient of the algorithm, which avoids the introduction of false information. The NLM algorithm is simple in theory and easy to be improved, and it can retain the information about the texture and structure of images well and effectively filter noises. Based on the advantages, considerable effects are obtained in many scientific research results. Tasdizen (2009) [24] analyzed NLM and principal component to reach the separation of image information from noise. As a result, the antinoise ability of the algorithm was significantly improved. Euclidean distance was changed, and a cosine function was introduced to improve the traditional NLM algorithm, which was then applied in the ultrasonic imaging intelligent diagnosis of localized scleroderma patients. SWE images of LS patients were assessed, and the improved NLM algorithm showed excellent denoising effects on LS patients' ultrasonic images. Skin high-frequency ultrasound technology is a new diagnostic technology. The physical characteristics of ultrasound can detect the whole layer of skin and skin accessories and can assist in the diagnosis of a variety of skin diseases, such as some pigmentation, skin aging, scleroderma, and the process of wound healing [25]. Seidenari et al. (2000) [26] showed that skin thickness increases with age. The changes in skin thickness, the thickness of skin dermis, and the synthesis of total collagen also increased significantly in the 3–5 years of life. Two-dimensional ultrasonic SWE was applied by Huang et al. to evaluate the characteristics of soft tissue, and the shear-wave signals with different subvolumes were aligned in the time direction to correct the time delay from continuous pulse-echo events. Then, the three-dimensional local frequency estimation algorithm was used for three-dimensional velocity reconstruction. The technology was verified on liver fibrosis models with different hardness, showing the most advanced SWE system. The proposed technique relied on low volume ratio imaging and could be implemented on widely available clinical ultrasound scanners. In this study, high-resolution ultrasound combined with SWE imaging technology was used to quantitatively evaluate the thickness of scleroderma. The results indicated a good effect. NLM denoising algorithm was introduced in the imaging process to intelligently denoise the formed ultrasonic image to make the image clearer. The comparison of skin thickness in different parts is illustrated in Figure 8. The skin thickness of the abdomen, chest, and left finger of the two groups was compared, respectively. The results showed that there was a significant difference between the LS group and the control group (*P* < 0.05).

The article "The Value of High-Resolution Ultrasound Combined with Shear-Wave Elastography under Artificial Intelligence Algorithm in Quantitative Evaluation of Skin Thickness in Localized Scleroderma" was published in 2022. Journal: Comput Intell Neurosci.

## 5. Conclusion

In this study, the NLM noise reduction algorithm is applied to the skin thickness diagnosis of patients with localized scleroderma, which effectively improves the efficiency of image feature extraction and classification. This study shows that ultrasonic elastic imaging has a certain value for the quantitative evaluation of skin thickness. The application of the NLM algorithm in high-resolution ultrasound combined with shear-wave elastic imaging has the effect of noise reduction and has a certain reference value in the clinic. However, in practical application, there are still some shortcomings. For example, the experimental data cannot completely eliminate the interference of subjective factors. Therefore, various indicators can be standardized. The number of samples in this study is small. In the future, more physiological and clinical data are expected to be added to further expand the sample research support [27].

## Figures and Tables

**Figure 1:** Classification and summary of ultrasonic elastography methods.

**Figure 2:** Schematic diagram of improved NLM algorithm.

**Figure 3:** Comparison of ultrasonic noise reduction images before and after the algorithm.

**Figure 4:** Quantitative evaluations of NLM algorithm denoising before and after improvement. (a–c) The results of MSE, PSNR, and SSIM, respectively.

**Figure 5:** Ultrasonic diagrams.

**Figure 6:** Comparison of elastic modulus values of SWE imaging “shell”.

**Figure 7:** ROC curve of shell taking 1mm elastic modulus.

**Figure 8:** ROC curve of 2mm elastic modulus taken by shell.

**Figure 9:** Comparison of skin thickness between two groups. *Note.*^*∗*^ indicates *P* < 0.05, and the difference was significant.

**Table 1:** Comparison between the critical value of elastic modulus of SWE imaging “shell” and AUC.

Shell	1mm			2mm		
	*E*_max_	Emean	Esd	*E*_max_	Emean	Esd
Auc	0.984	0.926	0.965	0.998	0.968	0.997
Threshold (KPa)	>88.97	>25.93	>18.69	>97.85	>28.67	>19.28

**Table 2:** Statistical results of LS lesions.

	Subjects (96 lesions)		
Different periods	Edema stage	Sclerotic stage	Atrophic stage
Number of lesions	7 cases	42 cases	47 cases
Proportion	7.29%	43.75%	48.96%

## Data Availability

The data used to support the findings of this study are available from the corresponding author upon request.
